# lncRNA Vgll3 Regulates the Activated Proliferation of Mouse Myocardial Fibroblasts through TGF-*β*3-Related Pathway

**DOI:** 10.1155/2022/2055738

**Published:** 2022-08-21

**Authors:** Bing Liu, Miao Chen, Wei Meng

**Affiliations:** ^1^Department of Emergency, Beijing Friendship Hospital, Capital Medical University, 100050 Beijing, China; ^2^Department of Cardiology, Beijing Friendship Hospital, Capital Medical University, 100050 Beijing, China

## Abstract

**Background:**

Cardiac fibrosis is a risk factor leading to various cardiac diseases, and its mechanism has not been clarified. However, long noncoding RNA (lncRNA) can mediate the pathological process of cardiac fibrosis.

**Objective:**

This study is aimed at determining the pathological role of lncRNA Vgll3 in cardiac fibrosis and explore its potential mechanism.

**Methods:**

Myocardium fibroblasts (CFs) were isolated from mice and stimulated with angiotensin II (Ang-II). The expression of Vgll3 and transforming growth factor-*β*3 (TGF-*β*3) were detected by real-time fluorescence quantitative PCR (qPCR). Double luciferase reporter gene and western blot analysis (WB) were used to detect the effect of Vgll3 on TGF-*β*3 expression. The qPCR and WB were used to detect TGF-*β*3 pathway markers such as TGF-*β*3 and SMAD4, as well as cardiac fibrosis markers such as *α*-smooth muscle actin (*α*-SMA), fibronectin (Fn), and type I collagen (Col1). The proliferation of CFs in mice was analyzed by Cell Counting Kit-8 (CCK8) and 5-bromo-2-deoxyuracil (EdU) method.

**Results:**

Upregulation of Vgll3 promoted the expression of TGF-*β*3 and its downstream molecules in mouse CFs, while silencing of Vgll3 inhibited the TGF-*β*3 pathway. Upregulation of Vgll3 significantly promoted the activation and proliferation of mouse CFs cells. It promoted the mRNA and protein levels of *α*-SMA, Fn, Col1, and Col3, while silencing the expression of Vgll3 had the opposite effect. The above effects of upregulation of Vgll3 were counteracted by TGF-*β*3 knockdown intervention.

**Conclusion:**

Vgll3 can promote the activation and proliferation of CFs in mice by activating TGF-*β*3-related pathway.

## 1. Introduction

Cardiac fibrosis will affect the systolic and diastolic function of the heart, leading to the occurrence of most heart diseases [1, 2]. Its pathological mechanism is related to the hyperactivity of cardiac fibroblasts (CFs), which may lead to the accumulation of extracellular matrix proteins, thereby negatively threatening cardiac structure and function [3]. In addition, CFs are also an essential mediator of acute and chronic fibrotic responses to stress caused by pathological processes such as myocardial infarction, hypertension, and tissue repair [4]. The activation of CFs promotes the fibrotic response by secreting key fibrotic mediators and shows an excessive increase in proliferation levels [5, 6]. Among them, mediators related to cardiac fibrosis include transforming growth factor-*β* (TGF-*β*) and platelet-derived growth factor [7]. Although more and more researchers have made great efforts to slow the progression of cardiac fibrosis, the molecular mechanism has not been clarified yet [8]. Further exploration and research on the containment of cardiac fibrosis are of great significance for the cognition, prevention, and treatment of cardiac fibrosis-related diseases.

Long noncoding RNA (lncRNA) is a regulatory medium for various biological events. It influences biological processes through chromatin modification and transcriptional and posttranscriptional processes [9]. lncRNA has been reported to be closely related to various cardiovascular diseases and can participate in regulating cardiac fibrosis pathological process and play a promoting or inhibiting role [10]. lncRNA Vgll3 is a lncRNA which plays a significant role in various cardiovascular diseases. lncRNA N379519 can promote cardiac fibrosis after infarction by targeting mir-30 [11]. lncRNA metastatic record of lung adenocarcinoma 1 (MALAT1) can promote cardiac fibrosis and worsen cardiac function after myocardial infarction by regulating TGF-*β*1 activity [12]. lncRNA myosin heavy chain-associated RNA transcripts (MHRT) can promote cardiac fibrosis after myocardial infarction by targeting mir-3185 and further enhancing myocardial collagen deposition and fibrosis [13]. In addition, some lncRNA members have anticardiac fibrosis effects. For example, the expression of lncRNA GAS5 in cardiac fibrosis tissues is significantly inhibited. Its restoration can effectively inhibit the excessive proliferation of CFs and thus inhibit the development of cardiac fibrosis [14]. lncRNA fibroblast growth factor 9-related factor (FAF) is also an anticardiac fibrosis regulator, which can prevent the pathological progression of cardiac fibrosis by targeting fibroblast growth factor 9 (FGF9) in CFs and inactivating TGF-*β*1-P-SMad2/3 signal transduction pathway [15]. TGF-*β*3 is an essential factor for cardiovascular development, which has been confirmed to mediate the pathological process of cardiac diseases such as cardiomyopathy and can regulate the development process of renal fibrosis, peritoneal fibrosis, and cardiac fibrosis in mice together with lncRNA [16, 17].

In this study, we first explored the functional role and potential mechanism of Vgll3 as a member of lncRNA in cardiac fibrosis. Vgll3 mainly plays a role in promoting cardiac fibrosis and can regulate the activation and proliferation process of CFs by TGF-*β*3-related pathways. Our study will provide new insights into the treatment of cardiac fibrosis-related diseases.

## 2. Materials and Methods

### 2.1. Experiments on Animals

This study has been approved by the Ethics Committee of Beijing Friendship Hospital, and animal experiments are conducted strictly following animal care guidelines. Forty newborn mice (Beijing Weitong Lihua Experimental Animal Technology Co., Ltd., C57BL6/J) were purchased and reared under 21 ± 2°C, 55% humidity, and 12 h light/dark cycle. Mice were placed in a sealed isoflurane chamber and treated with isoflurane (2% V/V, flow rate 0.6 L/min; Shanghai YJ Biotechnology Co., Ltd., YJ-20946R). The mice were placed on wet ice approximately 30 seconds later to induce hypothermia anesthesia. The mouse ventricular vertices were collected, and the primary cells were separated by trypsin digestion and differential centrifugation. Finally, the mice were sacrificed by cervical dislocation.

### 2.2. Cell Culture and Transfection

We isolated mouse CFs using type I collagenase (Jiangsu Qi Biotechnology Co., Ltd., 2-0004) and cultured the CFs in Dulbecco modified Eagle medium (Shanghai Limai Bioengineering Co., Ltd., LM-P0523) containing 10% fetal bovine serum at 37°C and 5% CO_2_. CF activation was induced by angiotensin-II (10-5 mm) (Shanghai Jizhi Biochemical Technology Co., Ltd., V48000-10 mg).

Lipofectamine® 2000 (Shanghai Yinjin Biotechnology Co., Ltd., 11668-019) was used to transfect cells. After transfection for 6 h, the medium was replaced with fresh medium. The transfections mainly included Vgll3-overexpressed plasmid and its control (Vgll3 and vector), TGF-*β*3-overexpressed plasmid and knockdown plasmid (TGF-*β*3 and SI-TGF-*β*3), and Vgll3 knockdown plasmid and its control (Si-VGLL3 and Si-NC). They are designed and synthesized by Hanhang Science & Technology (Shanghai) Co., Ltd.

### 2.3. Real-Time Fluorescence Quantitative PCR (qPCR)

Total RNA was isolated from cultured mouse CFs using TRIzol reagent (Beijing Bioolebo Technology Co., Ltd., BTN81027-UJE). Then, total RNA (0.5 *μ*g) was reverse-transcribed using a cDNA reverse transcription kit (Shanghai Yanhai Biotechnology Co., Ltd., F-K1622) to obtain cDNA. RNA levels of Vgll3, TGF-*β*3, SMAD2, SMAD4, *α*-smooth muscle actin (*α*-SMA), fibronectin (Fn), and type I collagen (Col1) were detected by ABI 7500 rapid real-time PCR system. Determined by SYBR Green I incorporation method with *β*-actin as internal reference.

### 2.4. Double Luciferase Activity Assay

We used the double luciferase reporter gene detection kit (Nanjing Novizan Biotechnology Co., Ltd., DD1205-01/02) for luciferase reporter gene detection. First, CFs transfected with TGF-*β*3 luciferase plasmids and Renilla luciferase plasmids (control plasmids) were treated with Vgll3-overexpressed plasmids or si-vgll3 for 48 h cleaved for 20 min at room temperature. The lysate was then incubated with luciferase detection reagent I, and absorbance was immediately collected at all wavelengths. Stop & Glo reagents were added to reread the absorbance of the plate. The first reading was TGF-*β*3 luciferase, and the second reading was Renilla luciferase (control luciferase). Luciferase activity is calculated by the ratio of the two readings.

### 2.5. Western Blot/Blotting (WB)

Total protein was extracted from CFs by RIPA buffer (Shanghai Yuanmu Biotechnology Co., Ltd., YZ-S0696Q). Protein concentration was measured using the Bradford Protein Assay kit (Shanghai Yubo Biotechnology Co., Ltd., YB80814-100). The same amount of protein was isolated and transferred to the PVDF membrane by 10% SDS-PAGE (Shanghai Xinyu Biotechnology Co., Ltd., XYX6011). Seal the film with 5% skim milk at room temperature for 1 h. Then, the western blots were detected with TGF-*β*3, SMAD2, SMAD4, *α*-SMA, Fn, Col1, and GAPDH primary antibodies at the dilution ratio of 1 : 2,000. GAPDH is used as an internal reference. Chemiluminescence signals were captured by the EasySee Western Blot kit (Shanghai Hengfei Biotechnology Co., Ltd., L00205C-1) and analyzed by ImageJ 1.43.

### 2.6. Cell Counting Kit-8 (CCK-8) Is Used to Measure Cell Viability

We used the CCK-8 kit (Beijing Corina Biotechnology Co., Ltd., R2740) to inoculate CFs at a 2 × 10^3^/well density in 96-well plates. 10 *μ*L CCK-8 was added to each well and incubated at 37°C for 2 h. The optical density (OD) values of CFs at 0 h, 24 h, 48 h, and 72 h were recorded at 450 nm by a full-wavelength microporous plate analyzer (Hangzhou Ao-Sheng Instrument Co., Ltd., AS-19010-00).

### 2.7. EdU Measures Cell Proliferation

EdU incorporation Detection kit (Shanghai Liumai Bioengineering Co., Ltd., LM0078L) was used to measure the proliferation ability of CFs. The proliferating cells doped with EdU showed green fluorescence, and the nuclei stained with DAPI for 10 min at 25°C showed blue fluorescence. The ratio of EdU-positive cells (green cells) to a total number of DAPI-positive cells (blue cells) was recorded.

### 2.8. Statistical Analysis

SPSS 23.0 was used for data analysis in this study. All data are expressed as mean ± standard deviation. Student's *T*-test was used to compare intragroup means, while one-way ANOVA was used to compare means among groups. *P* < 0.05 is considered a statistically significant difference.

## 3. Results

### 3.1. Vgll3 Promoted the Expression of TGF-*β*3 in Mouse CFs

First, we investigated the transfection efficiency of Vgll3-overexpressed plasmid and inhibitory plasmid, and the data showed that both realized upregulation or downregulation of Vgll3 expression (Figures 1(a) and 1(b)). TGF-*β*3 mRNA expression level of mouse CFs was significantly increased when transfected with Vgll3-overexpressed plasmid, while the TGF-*β*3 mRNA expression level of mouse CFs was significantly decreased when transfected with Vgll3-inhibited plasmid (Figures 1(c) and 1(d)). In the dual-luciferase reporter gene assay, the overexpressed plasmid Vgll3 could significantly induce the luciferase activity of TGF-*β*3, while the knockdown of Vgll3 could significantly inhibit the luciferase activity of TGF-*β*3 (Figures 1(e) and 1(f)). WB analysis also showed that upregulation of Vgll3 significantly promoted the secretion of TGF-*β*3 protein, while downregulation of Vgll3 significantly inhibited the expression of TGF-*β*3 protein (Figures 1(g) and 1(h)). Vgll3 positively regulated the expression of TGF-*β*3, a key profibrotic factor.

### 3.2. Vgll3 Regulates Protein and mRNA Levels of the TGF-*β*3 Signaling Pathway

To further understand the underlying mechanism of TGF-*β*3 regulation by Vgll3, we analyzed its effect on the TGF-*β*3 pathway. The results showed that mRNA levels of TGF-*β*3 (Figure 1(c)), SMAD2, and SMAD4 pathway markers were significantly upregulated after transfection of Vgll3-overexpressed plasmid (Figure 2(a)). The mRNA levels of TGF-*β*3 (Figure 1(d)), SMAD2, and SMAD4 (Figure 2(b)) were significantly inhibited by transfection of Vgll3 inhibitory plasmid. WB detection and upregulation of Vgll3 significantly promoted the protein levels of TGF-*β*3 (Figure 1(g)), SMAD2, and SMAD4 (Figure 2(c)), while knockdown of Vgll3 significantly inhibited the protein levels of TGF-*β*3 (Figure 1(h)), SMAD2, and SMAD4 (Figure 2(d)).

### 3.3. Vgll3 Can Regulate the Activation of CFs in Mice

We assessed the effect of Vgll3 on CF activation in mice by detecting cardiac fibrosis markers. The results showed that overexpression of Vgll3 could significantly increase the mRNA levels of *α*-SMA, Fn, and Col1 (Figure 3(a)) and significantly promote the protein levels of these three indicators (Figure 3(c)). In addition, knockdown of Vgll3 also significantly inhibited *α*-SMA, Fn, Col1 mRNA, and protein levels (Figures 3(b) and (d)).

### 3.4. Vgll3 Could Regulate the Proliferation of CFs in Mice

We also evaluated the effect of Vgll3 on the proliferation of CFs in mice by the CCK8 method and EdU method. Data showed that Vgll3-overexpressed plasmid could significantly promote the proliferation ability of mouse CFs (Figures 4(a) and 4(c)) and increase the percentage of EdU active cells in mouse CFs (Figure 4(e). However, knockdown of Vgll3 significantly reduced the proliferation ability of CFs and the percentage of EdU active cells in mice (Figures 4(b), 4(d), and 4(f)).

### 3.5. In Mouse CFs, Vgll3 Regulates Cell Activation and Proliferation through TGF-*β*3-Related Pathways

In order to further explore the regulatory mechanism of Vgll3 on the activation and proliferation of CFs in mice, we conducted a further study. First, we found no significant difference in the influence of Vgll3+SI-TGF-*β*3 on the expression of Vgll3 compared with that of Vgll3-overexpressed plasmid alone, indicating that SI-TGF-*β*3 did not reverse the expression of Vgll3 (Figure 5(a)). However, Vgll3+SI-TGF-*β*3 intervention significantly offsets the influence of Vgll3 overexpression on TGF-*β*3 and *α*-SMA mRNA levels (Figure 5(a)) but also offsets the promotion of Vgll3 overexpression on CF proliferation and EdU active cell percentage in mice (Figures 5(a), 5(c), and 5(e)). In addition, compared with si-VGLL3 alone, si-VGLL3+TGF-*β*3 intervention had no significant effect on Vgll3 mRNA level in mouse CFs (Figure 5(b)). However, si-VGLL3+TGF-*β*3 intervention could reverse the inhibitory effect of Vgll3 knockdown on TGF-*β*3 and *α*-SMA mRNA (Figure 5(b)) and reverse the inhibitory effect Vgll3 knockdown on CF proliferation ability and EdU active cell percentage (Figures 5(d) and 5(f)).

## 4. Discussion

Cardiac organ injury will activate complex biological cascade reactions, leading to cardiac fibrosis [18]. Cardiac fibrosis may eventually lead to heart failure in the body, the leading cause of morbidity and mortality worldwide [19]. lncRNAs can influence gene expression through epigenetic effects, selective splicing, or acting as molecular sponges to play a role in biological development or disease progression and mediate cardiac fibrosis, which may become therapeutic targets for cardiovascular diseases [20]. Vgll3 may serve as a potential therapeutic target for cardiac fibrosis in this study.

TGF-*β*3 belongs to the multifunctional peptide superfamily, which can regulate cell growth and differentiation and play a particular role in tissue fibrosis [21]. It is known that it can induce cell-specific transcription programs by regulating SMAD signal transduction pathways, thus affecting the biological behavior of cells [22]. Studies have shown that TGF-*β*3 is significantly upregulated in human myocardial infarction tissues. Its expression increases significantly with the development of fibrosis after myocardial infarction, suggesting that TGF-*β*3 may be a driving factor in cardiac fibrosis [23]. Our observations showed that Vgll3 positively regulated mRNA and protein expression of critical profibrotic factor TGF-*β*3. Specifically, overexpression of Vgll3 significantly promoted mRNA and protein expression of TGF-*β*3, while knockdown of Vgll3 significantly inhibited mRNA and protein expression of TGF-*β*3. Our luciferase reporter gene assay also confirmed that Vgll3 positively regulates TGF-*β*3 transcription. Some previous studies have confirmed that lncRNA can affect the process of cardiac fibrosis and other diseases by regulating the transcription of some proteins. For example, lncRNA H19 can negatively regulate the expression of DUSP5 and affect the proliferation and fibrosis of CFs. lncRNA homeoframe A11 antisense (HOXA11-AS) can promote the growth and metastasis of CFs through positive regulation of TGF-*β*1, thus worsening the process of cardiac fibrosis [24, 25].

The pathological process of cardiac fibrosis involves the activation and proliferation of CFs [26]. In this study, cardiac fibrosis markers such as *α*-SMA, Fn, and Col1 were used to evaluate the activation of CFs [27], and the proliferation capacity of CFs was evaluated by CCK8 and EdU methods. In our study, the mRNA and protein levels of *α*-SMA, Fn, and Col1 were significantly increased under Vgll3-overexpressed plasmid. In contrast, the levels of these indicators were significantly inhibited under si-VGLL3 intervention, suggesting that Vgll3 can promote the activation of CFs in mice. In terms of proliferation, we found that overexpression of Vgll3 could significantly promote the proliferation of CFs in mice and increase the percentage of EdU active cells. In contrast, the knockdown of Vgll3 showed a significant opposite effect, suggesting that Vgll3 could positively regulate the proliferation of CFs in mice. In order to understand the underlying mechanism of Vgll3 in cardiac fibrosis, we further studied it. Our study showed that the promotion effect of Vgll3 overexpression on the activation and proliferation of CFs in mice could be counteracted by TGF-*β*3 knockdown. This suggests that Vgll3 in mouse CFs affects CF activation and proliferation by regulating TGF-*β*3-related pathways.

Although our study confirmed that Vgll3, as a member of lncRNA, can promote cardiac fibrosis by activating TGF-*β*3-related pathways, our study still has some limitations and needs further improvement. First, we can analyze the downstream miRNAs related to Vgll3 to further improve the molecular pathways related to the influence of Vgll3 on cardiac fibrosis. Secondly, we can supplement animal studies to further analyze the effects of Vgll3 on animal cardiac function and CFs in vivo. We will gradually improve around these aspects in the future.

## 5. Conclusion

In this study, our data suggest that Vgll3 positively regulates CF activation and proliferation in mice by activating TGF-*β*3-related pathways. We proved for the first time that Vgll3, as a driver of cardiac fibrosis, has targeted therapeutic potential, and targeted knockdown of cardiac fibrosis may play a specific anticardiac fibrosis therapeutic role, providing new insights into the molecular mechanism and treatment of cardiac fibrosis.

## Figures and Tables

**Figure 1:** Vgll3 promotes TGF-*β*3 expression in mouse CFs. (a and b) QPCR was used to detect the transfection efficiency of Vgll3-overexpressed and knockdown plasmid. (c and d) QPCR was used to detect the effects of Vgll3-overexpressed plasmid and knockdown plasmid on TGF-*β*3 expression in mouse CFs. (e and f) Effects of Vgll3-overexpressed plasmid and knockdown plasmid on TGF-*β*3 relative luciferase activity in mouse CFs were detected by double luciferase activity assay. (g and h) WB was used to detect the influence of Vgll3-overexpressed plasmid and knockdown plasmid on TGF-*β*3 protein level. Note: compared with control, ^∗∗^*P* < 0.01.

**Figure 2:** Vgll3 regulates protein and mRNA levels of the TGF-*β*3 signaling pathway. (a and b) QPCR was used to detect the effects of Vgll3-overexpressed plasmid and knockdown plasmid on TGF-*β*3 pathway markers. (c and d) Effects of Vgll3-overexpressed plasmid and knockdown plasmid on TGF-*β*3 pathway markers were detected by WB. Note: compared with control, ^∗∗^*P* < 0.01.

**Figure 3:** Vgll3 regulates the activation of CFs in mice. (a and b) The qPCR was used to detect the effects of Vgll3-overexpressed plasmid and knockdown plasmid on *α*-SMA, Fn, and Col1. (c and d) WB detected the effects of Vgll3-overexpressed and knockdown plasmid on *α*-SMA, Fn, and Col1. Note: compared with control, ^∗^*P* < 0.05 and ^∗∗^*P* < 0.01.

**Figure 4:** Vgll3 can regulate the proliferation of CFs in mice. (a and b) Effects of CCK8 on the proliferation of CFs in mice by detecting Vgll3-overexpressed plasmid and knockdown plasmid. (c and d) Effects of transwell on the proliferation of CFs in mice by detecting Vgll3-overexpressed and knockdown plasmid. (e and f) EdU detected the effect of Vgll3-overexpressed plasmid and knockdown plasmid on the proliferation of CFs in mice. Note: compared with control, ^∗∗^*P* < 0.01.

**Figure 5:** Vgll3 in mouse CFs regulates cell activation and proliferation through TGF-*β*3-related pathways. (a and b) QPCR was used to detect the effects of Vgll3+SI-TGF-*β*3 or SI-VGLL3+TGF-*β*3 on Vgll3, TGF-*β*3, and *α*-SMA. (c and d) CCK8 was used to detect the effects of Vgll3+SI-TGF-*β*3 or Si-VGLL3+TGF-*β*3 on the proliferation of CF cells. (e and f) EdU detected the effects of Vgll3+Si-TGF-*β*3 or Si-VGLL3+TGF-*β*3 on the proliferation of CFs cells. Note: compared with control, ^∗∗^*P* < 0.01.

## Data Availability

The data used to support the findings of this study are available from the corresponding author upon request.
